# The development of salt-sensitive hypertension regulated by PSGL-1 gene in mice

**DOI:** 10.1186/s13578-018-0218-2

**Published:** 2018-03-07

**Authors:** Yuhui Yang, Xue Liu, Yunpeng Liu, Hui Fu, Ying Gao, Xing Liu, Xiaoliang Jiang

**Affiliations:** 1 Beijing No. 8 High School. 2 Xue Yuan Street, Xicheng District, Beijing, 100032 People’s Republic of China; 2 Institute of Laboratory Animal Science, Chinese Academy of Medical Sciences (CAMS) & Comparative Medicine Centre, Peking Union Medical Collage (PUMC), 5 Pan Jia Yuan Nan Li, Chaoyang District, Beijing, 100021 People’s Republic of China

**Keywords:** PSGL-1, Salt-sensitive hypertension, Inflammation

## Abstract

**Background and objective:**

Chronic inflammatory is involved in the development of salt-sensitive hypertension and other cardiovascular diseases. PSGL-1 plays an important role in the inflammatory response.

**Methods and results:**

In this study, we used PSGL-1^−/−^ and PSGL-1^+/+^ mice fed with high salt diet to measure the blood pressure, inflammatory response and vascular injury. We found that, in PSGL-1^+/+^ mice, high salt diet resulted in high blood pressure with the increased expression of serum inflammatory cytokines IL-6, IL-1β and TNFɑ, vascular injury markers MCP-1, ET-1, and VWF, and renal macrophages and T cells infiltration, and endothelium-dependent acetylcholine vasodilation dysfunction. However, the influence was not found in PSGL-1^−/−^ mice. The deficiency of PSGL-1 prevented the increased adhesion of peripheral blood mononuclear cells to endothelial cells by high salt environment.

**Conclusions:**

Our results indicate that PSGL-1 is involved in the development of salt-sensitive hypertension via vascular inflammation and injury. The high salt induced inflammation may be initiated by leukocytes and endothelial cells adhesion through PSGL-1 binding with P-selectin or/and E-selectin.

## Background

Epidemiological and experimental studies have demonstrated a close relationship between salt intake and hypertension [1]. It has been estimated that 30–50% of hypertensive humans are salt-sensitive and at least 25% of normotensive individuals also show salt sensitivity [2]. Salt-sensitivity confers an increased risk for the occurrence of hypertension, and for cardiovascular disease such as stroke, coronary heart disease, cardiac insufficiency, and kidney disease [3]. Although the etiology of salt-sensitive hypertension is actually multifactorial, including vasoconstriction and retention of renal sodium/water metabolism, but the blood pressures of a considerable proportion of patients with hypertension can not be effectively controlled by vasodilators and diuretics [4]. In recent years, it has been reported that chronic inflammatory reaction is involved in the development of salt-sensitive hypertension and other cardiovascular diseases [5]. The inflammatory reaction and vascular injury may be an important mechanism of salt-sensitive hypertension and target organ injury [6].

P-selectin glycoprotein ligand-1 (PSGL-1), a transmembrane glycoprotein expressed on circulating leukocytes, and participates in leukocyte recruitment and lymphocyte homing as a major selectin ligand. PSGL-1 can significantly enhance platelet-activating factor-induced leukocyte activation, and interact with cytokines such as integrins to promote leukocyte adhesion [7]. Studies have shown that PSGL-1 is involved in the regulation of T lymphocyte differentiation process and its induced immune response. Inflammatory cytokines released by leukocytes, such as TNFα and IL-1, also can induce the adhesion between leukocyte PSGL-1 and selectins in endothelial cells or platelets, which promote the development inflammation [8]. Therefore, PSGL-1 plays an important role in the inflammatory response, but whether it is involved in the pathological development of salt-sensitive hypertension remains unknown. In order to detect the role and mechanism of PSGL-1 in the development of salt-sensitive hypertension, we used PSGL-1 knockout (PSGL-1^−/−^) and wild-type (PSGL-1^+/+^) mice fed with high salt diet to measure the blood pressure, inflammatory response and vascular injury.

## Methods

### Materials

The mouse brain endothelial cell line (Bend3) cells were purchased from Feng Hui Biological Technology Company (China). PSGL-1^+/+^ and PSGL-1^−/−^ mice were obtained from Department of Molecular Biology and Biochemistry, University of Oklahoma Health Science Center. Rabbit anti-mouse CD68 (ab955), and CD3 (ab16669) were purchased from Abcam (United Kingdom); Rabbit anti-mouse IL6 (21865-1-AP), TNFɑ (60291-1-Ig) were from Proteintech (United Kingdom). Mouse anti-IL1 (sc-130325) was from Santa Cruz Biotechnology Inc (Texas, USA.). ELISA Kits (BMS6002, KMC0061, EH3TNFA) were from Thermo Fisher. Phenylephrine (P1240000-1EA) and Acetylcholine chloride (PHR1546) were purchased from Sigma-Aldrich.

### PSGL-1^−/−^ mice and blood pressure measurement

PSGL-1^+/+^ and PSGL-1^−/−^ mice at 8 weeks were fed with low salt diet (0.4% NaCl) and high salt diet (6% NaCl) for 3 months. The blood pressures were measured from the aorta, via the left carotid artery, under isoflurane (1.5–2.5%, inhaled) anesthesia. The kidneys and blood samples were collected for immunofluorescence and ELISA. Thoracic aortas were collected for immunoblotting and vascular relaxation study.

### Enzyme-linked immunosorbent assay (ELISA)

Inflammatory cytokines TNF-α, IL-1β, and IL-6 in the serum from PSGL-1^+/+^ and PSGL-1^−/−^ mice were tested by ELISA Kits. Briefly, serum samples were added in the coated wells with TNF-α, IL-1β, and IL-6 mAb of 96-well plates and incubated for 1 h at room temperature, washed four times and then incubated with an HRP-linked streptavidin solution for 30 min at room temperature in the dark. All samples were tested by duplication, and absorbency was measured at 620 nm by a microplate reader (Sunrise Remote, Switzerland).

### Immunofluorescence staining

The kidneys of the mice were formalin-fixed, paraffin-embedded, and cut into 4-μm sections. Sections were deparaffinized with xylene and alcohol series, and antigen unmasking was performed through pressure cooker treatment in sodium citrate buffer. Sections were blocked using goat serum for 30 min at room temperature and then stained with antibodies against CD68 and CD3 respectively overnight at 4 °C, washed with PBS 3 times for 3 min each time. Sections next were incubated with Alexa Fluor 488 or 568 conjugated phalloidin. Fluorescent signals were captured using a confocal microscope.

### Vascular relaxation

Thoracic aortas were harvested from PSGL-1^+/+^ and PSGL-1^−/−^ mice, and placed in chilled buffer. The vessel rings were suspended in 5-mL organ baths containing oxygenated Krebs–Henseleit buffer (118 mM NaCl, 25 mM NaHCO3, 4.6 mM KCl, 1.2 mM MgSO4, 1.2 mM KH2PO4, 1.25 mM CaCl2, 10 mM glucose, 0.025 mM EDTA, PH 7.4 at 37 °C). After equilibration for 60 min, contractile responses were recorded. Aortic rings were exposed to a 100 μM KCl-depolaring solution and, after washout, they were then exposed to a range of concentrations of PE (10^−10^ to 10^−6^ mol/L). The functional integrity of this structure was confirmed by the dose response to Ach (10^−9^ to 10^−6^ mol/L).

### Immunoblotting

Mouse thoracic aortas homogenates were prepared for immunoblotting according to our previously published procedure [9] The samples were immunoblotted with well characterized anti-mouse MCP-1, ET-1, and VWF antibodies. Uniformity of protein loading and membrane transfer were determined by immunoblotting for GAPDH.

### Cell culture and adhesion test

The Bend3 cells were cultured with DMEM high glucose medium, supplemented with 10% fetal bovine serum, 100 μg/mL penicillin and 10 μg/mL streptomycin, and grown in 96-well plates treated with normal salt medium (133 mM) and additional 40 mM NaCl for 3 h. Peripheral blood mononuclear cells (PBMC) were isolated from PSGL-1^+/+^ and PSGL-1^−/−^ mice. Peripheral blood collected in EDTA-coated tubes was mixed with 1% methylcellulose and centrifuged at 25*g* for 15 min. The upper phase was then diluted with PBS to the original volume of blood/methylcellulose mixture, carefully layered onto a Histopaque 1.077 gradient and centrifuged at 250*g* for 30 min without brake. The PBMC-containing layer was collected, washed, and resuspended in RPMI-1640 medium for further incubation. The PBMC was stained with the ratio-fluorometric 2′,7′-*bis*-(2-carboxyethyl)-5-carboxyfluorescein acetoxymethyl ester (BCEC-F-AM) for 30 min at 37 °C, and then co-cultured with Bend3 cell for 30 min at 37 °C. Fluorescent signals were captured using a confocal microscope (Leica).

### Statistics

The data were expressed as mean ± SEM. Significant difference between two groups was determined by the Student’s *t* test. A value of P < 0.05 was considered statistically significant.

## Results

### PSGL-1 deficiency prevents the increased blood pressure induced by high salt intake

The blood pressure of PSGL-1^+/+^ mice fed with high salt diet was significantly higher than normal salt diet group. However, the increased blood pressure was not found in PSGL-1^−/−^ mice with high salt diet (Fig. 1), which means that PSGL-1 is involved in the development of salt induced hypertension.

**Fig. 1:** Systolic blood pressure in PSGL-1^+/+^ and PSGL-1^−/−^ mice. Systolic blood pressure was measured from the aorta, via the left carotid artery, under isoflurane anesthesia. *P < 0.05 versus PSGL-1^+/+^ with normal salt diet; ^#^P < 0.05 vs PSGL-1^+/+^ with high salt diet, *t* test, n = 6

### PSGL-1 deficiency inhibits the increased serum inflammatory cytokines expression by high salt intake

Vascular inflammation is closely related to salt sensitive hypertension, therefore we explored the expression of inflammatory cytokines in the serum of PSGL-1^+/+^ and PSGL-1^−/−^ mice. The serum levels of TNF-α, IL-1, and IL-6 were significantly elevated in PSGL-1^+/+^ mice with high salt diet compared with normal salt group. However, the increased expression of these inflammation cytokines was not observed in PSGL-1^−/−^ mice with high salt diet (Fig. 2).

**Fig. 2:** Serum levels of inflammatory cytokines in PSGL-1^+/+^ and PSGL-1^−/−^ mice with high salt or normal salt intake. Serum levels of TNF-α, IL-1β, and IL-6 were measured by ELISA kits. *P < 0.05 vs PSGL-1^+/+^ with normal salt diet; ^#^P < 0.05 versus PSGL-1^+/+^ with high salt diet, *t* test, n = 6

### PSGL-1 deficiency inhibits high salt-induced inflammatory cells infiltration

In order to further test the inflammation regulated by PSGL-1, we measured the number of macrophages and T cells in kidney tissue by immunofluorescence. We found that the number of macrophages (CD68) (Fig. 3a–d) and T cells (CD3) (Fig. 3e–h) in kidney were significantly increased after high salt intake than normal salt diet in PSGL-1^+/+^ mice, while the increased number of infiltrated inflammatory cells by high salt diet was not found in PSGL-1^−/−^ mice.

**Fig. 3:** The infiltrated macrophages and T cells in the kidney of PSGL1^+/+^ and PSGL1^−/−^ mice. **a**–**d** Macrophages infiltration in the kidney of PSGL1^+/+^ and PSGL1^−/−^ mice. **e**–**h** T cells infiltration in the kidney of PSGL1^+/+^ and PSGL1^−/−^ mice. MPO: Neutrophil; CD68: macrophage; CD3: lymphocyte

### PSGL-1 deficiency alleviates the high salt induced vascular dysfunction and injury

To examine the effect of PSGL-1 on vascular function injured by high salt diet, we measured ex vivo vascular function in PSGL-1^+/+^ and PSGL-1^−/−^ mice fed with high salt and normal salt diet respectively by recording concentration-relaxation curves using powerlab system. We found that high-salt diet resulted in endothelium-dependent acetylcholine (Ach) vasodilation dysfunction (Fig. 4a) and increased expression of vascular injury markers MCP-1, ET-1, and VWF in the thoracic aortas of PSGL-1^+/+^ mice (Fig. 4b). However these phenomenon was not found in PSGL-1^−/−^ mice.

**Fig. 4:** Regulation of PSGL-1 on high salt-induced vascular injury. **a** The vascular relaxation function was qualified by Powerlab system after Ach treatment. **b** The expression of vascular injury marker was quantified by immunoblotting in thoracic aortas of PSGL-1^+/+^ and PSGL-1^−/−^ mice. Results were corrected for expression of GAPDH protein. *P < 0.05 versus PSGL-1^+/+^ mice with 0.4% NaCl; ^#^P < 0.05 versus PSGL-1^+/+^mice with 6% NaCl, *t*-test, n = 6

### PSGL-1 deficiency inhibits high salt-induced leukocyte-endothelial adhesion

To detect of the mechanism of inflammation regulated by PSGL-1, we tested the leukocyte-endothelial adhesion by using PBMC and Bend3 cells co-culture system. We found that the number of PBMC (green color) from PSGL-1^+/+^ mice adhering to Bend3 cells was significantly increased in high salt medium (173 mM NaCl) than in normal saline medium (133 mM NaCl). The number of PBMC from PSGL-1^−/−^ adhering to Bend3 cells was not increased by high salt medium (Fig. 5), which indicates that PSGL-1 may play an important role in the high salt induced inflammation by regulating the adhesion of peripheral blood mononuclear cells to endothelial cells.

**Fig. 5:** The number of PBMC adhering to Bend3 cells co-cultured in normal and high salt medium. The Bend3 cells were co-cultured with PBMC from PSGL-1^+/+^ and PSGL-1^−/−^ mice stained with the ratio-fluorometric 2′,7′-bis-(2-carboxyethyl)-5-carboxyfluorescein acetoxymethyl ester (BCEC-F-AM) at normal salt (133 mM) and high salt (173 mM) medium. Fluorescent signals were captured using a confocal microscope (Leica). Green represents the number of adhered PBMC

## Discussion

In recent years, salt sensitive hypertension is considered to be a chronic inflammatory disease [5]. In this study, we found that high salt diet increased blood pressure in PSGL-1^+/+^ but not in PSGL-1^−/−^ mice. The increased blood pressure in PSGL-1^+/+^ mice with high salt diet was accompanied with increased expression of serum inflammatory cytokines IL-6, IL-1β and TNFɑ, and renal macrophages and T cells infiltration. IL-6, IL-1β and TNFɑ are mainly secreted by activated macrophages and T cells that play an important role in the development of inflammatory response [10]. TNFɑ stimulates endothelial cells to secrete other inflammatory factors and then promotes inflammation, and induces vasodilatory dysfunction by inhibiting the expression of eNOS [11]. The TonEBP-VEGF-C signaling in mononuclear phagocyte system (MPS) is involved in the development of salt-sensitive hypertension via vascular eNOS secretion [12]. Therefore, PSGL-1 is involved in the development of salt-sensitive hypertension via inflammation.

The main purpose of hypertension control is to prevent the target organ injury. It was found that PSGL-1-p-selectin interactions contributed to vascular injury and exacerbated atherosclerosis [13]. In this study, we found that high-salt diet caused endothelium-dependent acetylcholine vasodilation dysfunction and increased the expression of vascular injury markers MCP-1, ET-1, and VWF in PSGL-1^+/+^ mice, but not in PSGL-1^−/−^ mice. There is evidence shows that each domain of the PSGL-1 molecule plays crucial roles in leukocyte activation and promote leukocyte rolling and extravasation to vascular endothelial and continuously aggravate endothelial injury [14]. Our finding indicates that PSGL-1 may participate in the regulation of vascular injury via inflammation by high salt intake, which may be the meaningful target of hypertension prevention.

PSGL-1 is responsible for the initial step of the inflammation via mediating interactions with P-selectin and E-selectin expressed by endothelial cells to initiate the ‘capture and rolling’ step in the leukocyte–endothelial cell adhesion cascade [15]. In this study, we found that the block of PSGL-1 prevented the increased adhesion of PBMC to endothelial cells by high salt environment with Endothelial Cells/PBMC co-culture system. The E-selectin expression was increased in the mouse brain endothelial cell line (Bend3) with high salt medium culture [16]. The interaction of PSGL-1 with P-selectin on activated platelet promoted the formation of leukocyte-platelet aggregates that contribute to adhesion and infiltration of inflammatory cells [17]. We also found that platelet further increased the number of PBMC adhesion to endothelial cells in the Endothelial Cells/PBMC co-culture system with high salt medium (data not shown). The inflammation caused by high salt intake may be initiated by leukocytes and endothelial cells adhesion with or without platelet activation through PSGL-1 binding with P-selectin or/and E-selectin.

In conclusion, PSGL-1 plays an important role in the development of salt-sensitive hypertension via vascular inflammation and injury. The high salt induced inflammation may be initiated by leukocytes and endothelial cells adhesion through PSGL-1 binding with P-selectin or/and E-selectin. However, the mechanism remains to be further studied.

## Abbreviations

PSGL-1: P-selectin glycoprotein ligand-1
MAP: mean artery pressure
PBMC: peripheral blood mononuclear cells
MPS: mononuclear phagocyte system
Bend3: mouse brain endothelial cell line
Ach: acetylcholine
PE: phenylephrine
IL-1β: Interleukin 1β
TNFɑ: tumor necrosis factor α
IL-6: Interleukin 6
MCP-1: Monocyte Chemotactic Protein-1
ET-1: Endothelin-1
vWF: Von Willebrand factor
PBS: phosphate-buffered saline
DMEM: Dulbecco’s modification of Eagle’s medium Dulbecco
BCEC-F-AM: phorbol 12-myristate 13-acetate
SDS: sodium dodecyl sulfate
